The article "Clinical Observation of Anatomical and Visual Outcomes of Macular Hole after Inverted Internal Limiting Membrane Flap in Patients with Idiopathic Macular" was published in 2023. Journal: J Healthc Eng.

# Clinical Observation of Anatomical and Visual Outcomes of Macular Hole after Inverted Internal Limiting Membrane Flap in Patients with Idiopathic Macular

**DOI:** 10.1155/2023/5816473

**Published:** 2023-02-15

**Authors:** Yunda Zhang, Jie Li, Huifang Yue, Zhao Gao, Tao Ma, Xiaohong Gao, Zhigang Yuan, Gaiyun Li, Ximei Zhang

**Affiliations:** ^1^Department of Vitreoretinopathy, Shanxi Eye Hospital, Taiyuan, Shanxi, China; ^2^Shanxi Medical University, Taiyuan, Shanxi, China

## Abstract

**Objective:**

To investigate anatomical and visual outcomes of macular hole (MH) after inverted internal limiting membrane (ILM) flap technique for idiopathic macular hole (IMH).

**Methods:**

A total of 13 IMH cases diagnosed in Shanxi Eye Hospital between January 2015 and June 2016 were included in the study. All patients underwent vitrectomy combined with indocyanine green-assisted inverted ILM flap technique. The MH closure rate, best-corrected visual acuity (BCVA), changes of ellipsoid zone (EZ), and external limiting membrane (ELM) were examined before operation and one, three, and six months after operation. Furthermore, 488 nm fundus autofluorescence (FAF) and spectral domain optical coherence tomography (SD-OCT) were used to observe the dynamic changes in function of macular area after surgery.

**Results:**

One month after the surgery, the MH closure rate was 100% and the visual acuity (VA) was stable, with no recurrence. Additionally, the average logMAR BCVA before operation was 1.208 ± 0.158, and this value became 0.877 ± 0.105 one month after the operation, showing a significant decrease. Three months after surgery, the average logMAR BCVA was 0.792 ± 0.103, which was significantly lower than the level one month after the surgery but much higher than that six months after surgery (0.708 ± 0.131). Besides, the diameter of the EZ defect of the postoperative one month, three months, and six months was (1377.46 ± 198.65) *μ*m, (964.62 ± 336.26) *μ*m, and (817.08 ± 442.99) *μ*m, respectively. In postoperative one month, three months, and six months, the diameter of the ELM defect diameter was (969.62 ± 189.92) *μ*m, (649.92 ± 413.15) *μ*m, and (557.62 ± 412.50) *μ*m, respectively. The diameter of both EZ and ELM defects was significantly reduced with the passage of time after surgery.

**Conclusion:**

Inverted ILM flap technique can reconstruct macular anatomical structure and improve VA. This technique is effective for the treatment of IMH with large MH minimum diameter and base diameter.

## 1. Introduction

A macular hole (MH) is a retinal defect that appears in the internal limiting membrane (ILM) and extends to (but not include) the retinal pigment epithelium (RPE). The prevalence of the disease varies from 0.2% to 0.8% among the public [1]. Idiopathic MH (IMH), accounting for most of MH cases, is a common retinal disease with no clear etiologies and with no association with fundus lesion itself. IMH has a higher prevalence in the elderly and presents as a primary cause of their central visual impairment and visual degeneration [2, 3]. This disease has long been considered incurable until 1991 when Kelly and Wendel first applied vitrectomy to successfully cure IMH [4]. Subsequently, in 1997, Eckardt first introduced internal limiting membrane (ILM) peeling to improve the closure rate of MH [5]. Vitrectomy combined with ILM peeling has qualified as the standard surgical approach for full-thickness MH, which has achieved a closure rate of 90%–100% and a visual acuity (VA) improvement rate of 85% [6, 7]. The most important factors affecting postoperative IMH closure and visual recovery are the minimum diameters of IMH and base diameter. Patients with the minimum diameter of MH <300 *μ*m and base diameter <1000 *μ*m present a good prognosis [8], but larger values of these two parameters cause a low closure rate and poor prognosis and therefore have formed an obstacle that clinicians have been trying to solve.

In 2010, Michalewska et al. reported the application of inverted ILM flap technique to MHs with a diameter over 500 *μ*m [7] and its satisfactory efficacy in improving VA and closure rate of IMH and myopic MHs [7]. A large-scale comparative study found that the closure rate was 95.6% and 88.4% in patients with IMH >400 *μ*m and myopic MH after the application of the inverted ILM flap technique [9]. Compared with ILM implantation technology, inverted ILM flap technology can better restore the photosensitive layer and obtain better functional results. For larger MHs (>700 *μ*m), filling can not only rebuild the closed environment, but also help the recovery of the hole. However, a meta-analysis showed that in patients with large MHs, vitrectomy with an inverted ILM flap technique had a higher rate of anatomical closure than ILM dissection. The inverted ILM flap technique had better visual recovery at short-term follow-up, but no advantage was found in longer-term follow-up. For patients with larger MHs, the inverted ILM valve technique should be considered the first-choice conventional treatment. Therefore, more randomized controlled trials with larger sample sizes and longer follow-up are recommended to confirm the effectiveness of the inverted ILM flap technique.

Optical coherence tomography (OCT) can clearly show retinal microarchitecture and has become the dominant imaging method for the diagnosis of retinopathy as well as the confirmation of the anatomical success after surgery for IMH [10]. Studies have shown that spectral domain OCT (SD-OCT) delineated structural changes in the photoreceptor layer of the eye after surgical closure of IMH, including disruption of the ellipsoidal zone (EZ) and external limiting membrane (ELM) after surgical closure of IMH. However, only a few studies have evaluated the anatomical reconstruction of fovea centralis after using the inverted ILM flap technique in IMH patients and have pointed out recovery from ELM is a key structure feature associated with postoperative best-corrected VA (BCVA) [11].

We used the inverted ILM flap technique to treat refractory IMH patients with large MHs and then observed anatomical and visual outcomes of MHs, to provide better treatment and sufficient theoretical basis for the treatment of IMH.

## 2. Materials and Methods

### 2.1. Research Subjects

Inpatients who were diagnosed with IMH in Shanxi Eye Hospital between January 2015 and June 2016 were collected. Patients with minimal hole diameter >500 *μ*m and base diameter >1000 *μ*m were selected and included. However, patients with the following conditions were excluded: (1) patients with other ocular diseases such as myopia, glaucoma, age-related macular degeneration, and uveitis; (2) patients with a history of ocular surgeries; (3) patients without continuous follow-up data. General data of the included patients were recorded. Informed consent was obtained from all patients, and the study had gained the approval of the Ethics Committee of Shanxi Eye Hospital (SXYYLL20211028).

### 2.2. Operation Methods

All patients in this study were treated by the same surgeon. First, a routine 25-G vitrectomy was performed. The posterior vitreous membrane was peeled off after intravitreal injection of a small amount of triamcinolone acetonide. Then, ILM was treated with indocyanine green dye (0.05 mg/mL), and ILM around MH with a diameter of about two optic discs was removed. Superior ILM attached to the margins of MH was left in place, and subsequently, the remnant ILM was inverted upside-down to cover the MH. After air/liquid exchange, the eyes were filled with 14% of C_3_F_8_ gas. All patients underwent ultrasonic emulsification combined with posterior chamber intraocular lens implantation. After surgery, patients were kept in a face-down position for two weeks.

### 2.3. Evaluation Indexes

Before the operation and one, three, and six months after the operation, BCVA was detected, and all patients received a slit-lamp examination, SD-OCT (Spectralis OCT of Heidelberg Engineering, Germany), and 488 nm fundus autofluorescence (FAF) examination (HRA-II, Heidelberg Engineering, Germany). SD-OCT was used to scan and measure the minimum diameter of MH and the maximum base diameter before surgery, as well as the defect diameter of EZ and ELM.

### 2.4. Statistical Analysis

SPSS19.0 statistical software was adopted for statistical analysis in this study. The measurement data were expressed as mean ± standard deviation (Mean ± SD), and a *t*-test was used to compare the results from the two groups. *P* < 0.05 was taken as a statistically significant difference.

## 3. Results

### 3.1. Inverted ILM Flap Technique Significantly Improves Macular Hole in Patients with IMH

The average age of the patients was 65.769 ± 3.479. The patients were examined by SD-OCT and FAF before surgery and one, three, and six months after surgery. Before surgery, the inverted ILM flap and its underlying liquid cavity were visible in the MH, and a high intensity of the FAF signal was also observed (Figures 1(a) and 1(b)). One month after the surgery, the liquid cavity disappeared in the MH, while protuberances demonstrating a moderate signal and particles showing a high signal appeared. Besides, a new area with a low FAF signal was observed (Figures 1(c) and 1(d)). Three months after surgery, the moderate signal protuberances became larger and new low FAF signal areas were observed between high fluorescence signals (Figures 1(e) and 1(f)). Six months after surgery, the abovementioned protuberances disappeared in the MH, and the ELM, EZ, and RPE layer defects were shown; additionally, the area with a low FAF signal was enlarged (Figures 1(g) and 1(h)).

### 3.2. Inverted ILM Flap Technique Significantly Enhanced the Visual Acuity of IMH Patients

The postoperative BCVA and MH closure rate was calculated and analyzed in accordance with SD-OCT and FAF examination in a bid to evaluate the therapeutic effect of the inverted ILM flap technique. The results showed that the minimum diameter of MH before surgery was 680 *μ*m, base diameter 1072 *μ*m, and the logMAR BCVA 1.208 ± 0.158. While one month after the operation, MH closure rate was 100% accompanied with “U”-shaped or “V”-shaped healing, and the condition remained stable during the follow-up period without recurrence; the logMAR BCVA levels of patients were significantly reduced, with an average logMAR BCVA of 0.877 ± 0.105; defect diameter of EZ and ELM stood at (1377.46 ± 198.65) *μ*m and (969.62 ± 189.92) *μ*m, respectively. Three months after the operation, the average logMAR BCVA was 0.792 ± 0.103, the diameter of EZ and ELM defect was (964.62 ± 336.26) *μ*m and (649.92 ± 413.15) *μ*m, respectively; significant differences were found in such indexes between one month and three months after surgery. Six months after the operation, the average logMAR BCVA of all patients was 0.708 ± 0.131, and the diameter of EZ and ELM defect was (817.08 ± 442.99) *μ*m and (557.62 ± 412.50) *μ*m, respectively; significant differences were found in such indexes between three months and six months after surgery. In addition, FAF examination showed that the patient's preoperative fundus fluorescence was strong, while it turned into low signal six months after surgery (Figure 2), suggesting that the inverted ILM flap technique was effective in the treatment of IMH patients.

## 4. Discussion

MH <400 *μ*m can be categorized into grades I and II, and its closure rate climbs from 58% to more than 90% after applying different treatment techniques combined with vitrectomy [11, 12]. However, 44% of patients with MH >400 *μ*m still suffered from MHs opened after conventional vitrectomy combined with ILM peeling [13], thus frequently necessitating a second operation [7]. Refractory MHs usually include MHs >400 *μ*m, pathological myopia combined with macular splitting, MHs lasting more than six months and undergoing multiple surgeries, or MHs with extensive retinal detachment or proliferative vitreoretinopathy. IMH patients included in this study were scanned by SD-OCT and measured to have a minimum diameter >500 *μ*m and a base diameter >1000 *μ*m, which are clinically refractory MHs. These patients received vitrectomy combined with inverted ILM flap technique and 100% closure rate. Such outcomes may be attributable to the fact that peeling off part of ILM can relieve the tangential traction of ILM at the MH. In addition, the inverted ILM flap covering the MH allows the hole to form a closed cavity and thus promotes the absorption of fluid in the MH through the RPE cell pump function. The inverted ILM flap covering the MH also stimulates the proliferation of glial cells in the retina and on the surface of ILM and acts as a scaffold for cell proliferation [7, 14]. Collectively, the inverted ILM flap technique promotes the closure of MHs.

Intraoperative peeling of the ILM is beneficial in removing completely the contractile tissue attached to it, reducing the tangential traction around the hole, removing the scaffold for the proliferation of fibroblasts and RPE cells, preventing the generation of epiretinal membrane, and preventing recurrence. Minor damage during ILM peeling can stimulate Müller cell proliferation and promote hole healing. However, in patients with larger hole diameters, unhealed after ILM peeling, and high myopic macular holes, the hole closure after surgery is higher than low-discovery ILM flap surgery and can promote the healing of postoperative MH healing, increase the closure rate of postoperative hiatus with a diameter >400 *μ*m, and improve patient visual acuity. After ILM flap operation, the ILM in the hole will not act as a foreign body to hinder the closing process of the hole. On the contrary, it will provide a scaffold for glial cells and promote the proliferation of glial cells, thereby pulling the photoreceptor cells to move to the center of the hole, promoting the hole is closed. Therefore, for patients who face difficulty in closing the hole after routine vitrectomy combined with ILM peeling, it can be combined with ILM flap surgery at the same time during the operation.

FAF can reveal the content and distribution of lipofuscin in RPE cells in a noninvasive manner, reflecting the functional status of RPE and photoreceptor cells. In this study, it was shown that the patient presented low FAF signals after surgery. Nonetheless, according to FAF examination results one month after the surgery, it was found that the MH was not closed and ILM was still present, with low signal spots in the macular area in the affected eye; three months after the surgery, OCT showed localized protuberance with moderate signal intensity in the inner retina and particles with high signal intensity in the outer retina, while FAF demonstrated an expansion of the area with low signal intensity. Such imaging outcomes may be the result of glial cell proliferation along the ILM flap [15, 16]. Six months after the surgery, the abovementioned protuberance and the high signal particles decreased; additionally, we observed the defect of EZ and RPE layers. The possible reason for the dynamic changes may be that the inverted ILM flap technique stimulates the activation and proliferation of glial cells such as Müller cells along the scaffold provided by the flap, which assisted the repairing and reconstruction of the retina; this inverted ILM flap technique-caused process is found the most obvious from the third to the fourth month [17]. However, while Müller cells are activated and proliferated, retinal microglia may also be activated to exert phagocytic function and produce a large amount of inflammatory substances (such as TNF-a, IL-1*β*) and to exert toxic effects on retinal cells. Consequently, such activation can result in the inhibition of excessive proliferation of glial cells and damage RPE cells [18, 19].

The diameter of IMH constitutes an important factor affecting the closure rate and postoperative VA [20]. Currently, OCT is used clinically to measure different parameters of MH to predict the closure of MHs and recovery of VA, such as the minimum diameter of the hole, the base diameters, the height of the hole, the angle between the margin of the hole and the base, and the various formulas deduced hereinafter [21, 22]. As reported, the minimum diameter and base diameters were important factors affecting postoperative MH closure and visual prognosis [8]. On top of it, the two parameters are easy to measure and calculate. The visual prognosis was related to “U”-shaped MH healing, normal thickness of fovea centralis, and integrity of photoreceptor layer [23]. In this study, it was found that the defect diameter of both EZ and ELM after surgery had a tendency to decrease during follow-up, indicating the fact that retinal photoreceptors and retinal Müller cells were gradually recovered and retinal structure was increasingly reconstructed. In addition, this study also revealed a gradual decrease in logMAR BCVA over time in postoperative patients, indicating that VA was restored. The improvement of postoperative VA may be attributed to the proliferation of glial cells which facilitate the repositioning of photoreceptor cells in the central fovea [7].

## 5. Conclusion

Inverted ILM flap technique can increase the postoperative closure rate of IMH with a large diameter. Additionally, it acts to improve postoperative VA as well as reconstruct the retinal structure. Therefore, this technique can serve as an effective treatment for MH with large minimum diameter and the large base diameter. However, whether the indocyanine green-assisted inverted ILM flap technique leads to retinal cell damage still requires more observation and research studies.

## Figures and Tables

**Figure 1:** Effect of inverted ILM flap technique on macular hole in IMH patients. Ocular SD-OCT and FAF images of one patient before surgery (a, b), one month after surgery (c, d), three months after surgery (e, f), and six months after surgery (g, h). The green arrow indicates the location and direction of OCT scanning; yellow arrows indicate protuberance with moderate signal intensity; red arrow indicates particles with high signal intensity; and blue arrows represent new spots with low signal intensity.

**Figure 2:** Effect of the inverted internal limiting membrane flap technique on visual acuity in patients with IMH ocular SD-OCT scanning of one patient before surgery (a), one month after surgery (b), three months after surgery (c), six months after surgery (d), ocular FAF images of one patient before surgery (e), and six months after the surgery (f). Postoperative BCVA and MH closure rate before and after operation (g–i). Yellow arrows indicate protuberance with moderate signal intensity; red arrows denote the range of fluorescence intensity. ^*∗*^*P* < 0.05, ^*∗∗*^*P* < 0.01, and ^*∗∗∗*^*P* < 0.001.

## Data Availability

The data used to support the findings of this study are available from the corresponding author upon request.
